# Understanding Supply-Side Implementation Barriers Affecting Child Nutrition Outcomes in the Take-Home Ration Scheme: A Qualitative Study From Madhya Pradesh, India

This article has been retracted.

**DOI:** 10.7759/cureus.106307

**Published:** 2026-04-02

**Authors:** Arun Kokane, Harijith K R, Junaid Mushtaq, Nikita Rawat

**Affiliations:** 1 Community and Family Medicine, All India Institute of Medical Sciences Bhopal, Bhopal, IND

**Keywords:** child nutrition, child nutrition programs, food and nutrition, food supply chain, supplementary nutrition program

## Abstract

Background

Child undernutrition persists as a critical public health challenge across India despite the extensive infrastructure of the Integrated Child Development Services (ICDS) program; child undernutrition remains persistently high, especially in Madhya Pradesh, where stunting affects 35.5% of children. The Take-Home Ration (THR) component, intended to provide supplementary nutrition to women and young children, continues to underperform due to interconnected supply-chain, governance, and community-level challenges. This study aimed to examine supply-side implementation barriers and assess the current status of THR distribution and Social and Behaviour Change Communication (SBCC) activities under ICDS in Madhya Pradesh, India, from a multi-stakeholder perspective.

Methods

This qualitative, multi-method study combined Net-Map supply chain analysis and semi-structured key informant interviews with 15 stakeholders spanning state, district, block, and community levels in Hoshangabad district, Madhya Pradesh, India. Thematic analysis using Braun and Clarke's framework identified systemic barriers and adaptive practices across seven organisational hierarchies.

Results

Network mapping revealed that the State Nutrition Committee, manufacturing divisions, and Anganwadi Centres function as non-substitutable backbone actors whose dependencies create systemic vulnerabilities. Identified constraints included multi-tiered supply chains causing cumulative delays, prolonged government payment cycles restricting manufacturer capacity, and product-community misalignment between fortification requirements and taste acceptability. Additional barriers comprised weak inter-departmental coordination, limited frontline capacity, and inadequate community engagement due to opportunity costs and digital connectivity gaps. Locally generated adaptive solutions-such as product modifications and community recipe innovations-remained institutionally disconnected from higher governance systems.

Conclusion

Strengthening THR implementation requires a coordinated systems approach emphasising fiscal accountability, decentralised decision-making, and context-specific, culturally grounded social and behaviour change communication. Institutionalising mechanisms that integrate frontline-derived learning into policy adaptation is essential for achieving resilient nutrition program delivery and improved outcomes.

## Introduction

Child undernutrition is a significant public health challenge in India, as India accounts for nearly one-third of the global burden of stunting and wasting among children under five years of age [1]. Despite this, data from the National Family Health Survey (NFHS-5) reveal that Madhya Pradesh faces high nutritional challenges for children. Presently, the prevalence of stunting is at 35.5%, wasting at 19.3%, and underweight at 32.1% [2]. The Integrated Child Development Services (ICDS) scheme, which was launched in 1975, currently operates in about 1.4 million Anganwadi Centres (AWCs) nationwide, representing the most extensive integrated program for early childhood care and development ​[3].

The Take-Home Ration (THR) component of ICDS is implemented to provide ready-to-eat or ready-to-cook supplementary nutrition to children aged 6-36 months and pregnant and lactating women from vulnerable households [4]. Along with the THR distribution system, ICDS and SBCC strategies are implemented for improving feeding practices to enhance program utilisation [5]. ICDS services have expanded significantly over the past years, but some evaluations suggest that implementation challenges continue to limit the program's effectiveness in addressing child undernutrition ​[6].

Despite various changes and continuous research on the ICDS program improvement, significant implementation gaps remain in understanding the complex interplay between THR provision, SBCC strategies, and community feeding practices from the perspectives of diverse stakeholders across the implementation hierarchy [7]. The previous studies on the Take-Home Ration (THR) program have concentrated mainly on quantitative indicators or the perspectives of a single group of stakeholders. This narrow focus has limited the understanding of the complex challenges and opportunities within the THR system. Moreover, there is still little evidence on how current THR formulations and SBCC strategies fit with the actual feeding habits, household practices, and cultural preferences of families in rural areas.

This study sought to address existing knowledge gaps by employing a qualitative, multi-stakeholder approach to examine the implementation of the THR program in Madhya Pradesh. Specifically, it aimed to explore supply-side stakeholders' perspectives on operational, governance, and human resource challenges influencing the THR supply chain, as well as to assess the current status of THR distribution and SBCC activities under ICDS in Madhya Pradesh, India. The study had two specific objectives: (1) To explore supply-side stakeholders' perspectives on operational, governance, and human resource challenges influencing the THR supply chain; and (2) To assess the current status of THR distribution and SBCC activities under ICDS in Madhya Pradesh, India.

## Materials and methods

Study design and context

This qualitative study was conducted as the formative research component of a larger cluster randomised controlled trial (cRCT) examining the effectiveness of improved THR combined with behaviour change communication interventions to enhance nutritional outcomes for children across six states in India [8]. This qualitative research specifically identified supply-side implementation barriers and facilitators affecting the quality, utilisation, and effectiveness of the THR scheme in Madhya Pradesh. The study was conducted in Hoshangabad district, located in the central region of Madhya Pradesh, India. AWCs and associated administrative structures across two blocks in the district were purposively selected as study sites.

Study population and sampling strategy

Using purposive sampling with maximum variation, we recruited key informants representing all organisational levels from state-level policy formulation to community-level service delivery. The sampling framework was designed to capture diverse stakeholder perspectives on the challenges and facilitators of the THR supply chain. We recruited 15 key informants across seven distinct stakeholder categories: Anganwadi Workers (AWWs, n=8), Child Development Project Officers (CDPOs, n=2), District Program Officers (DPOs, n=1), State Program Officers (SPOs, n=1), THR Manufacturing Unit Managers (n=1), United Nations Children's Fund (UNICEF) Program Representatives (n=1), and Non Government Organizations (NGO) State Program Coordinators (n=1). Participants were eligible if they held direct or indirect responsibility for THR program planning, implementation, monitoring, or utilisation for ≥6 months at the time of data collection. The sample size of 15 was determined a priori based on the purposive maximum variation sampling strategy, designed to ensure representation across all seven stakeholder categories spanning the full implementation hierarchy. Rather than being guided by iterative saturation testing, the sampling framework prioritised comprehensive tier coverage to enable a systems-level perspective.

Data collection methods

Data collection was conducted over four months (April-August 2025) using a sequential two-step mixed-methods approach that combined supply chain mapping with in-depth qualitative interviews.

Step 1: Net-Mapping of THR Supply Chain

To systematically trace THR flows from policy formulation through distribution, net-mapping exercises were conducted in two separate sessions. The first session included four participants comprising district and block-level officials, and the second session included one state-level official. Using large sheets of paper and colour-coded markers (blue for information flows, red for financial flows, green for food commodity flows), participants identified all relevant actors from national-level policy bodies (e.g., the Secretary, Government of India) through to frontline workers and beneficiaries. The net-mapping protocol followed a structured five-step process: (1) mapping the supply chain flow; (2) identifying key actors at each stage; (3) clarifying the roles of each actor; (4) linking actors through directional arrows indicating the nature of the relationship (food, information, or financial flows); and (5) assessing influence through participatory scoring. Sequenced actors according to their formal roles, responsibilities, and organisational hierarchy. Mapped directional arrows indicating pathways and relationships for data, funds, and commodities. Influence scores were assigned using a 1-5 star rating scale based on pre-defined criteria: each actor's contribution to ensuring THR quality, timeliness of delivery, efficiency of fund transfer, and capacity for adaptive program management. These criteria were explained to participants prior to scoring. Ratings were assigned through facilitated group consensus, with the research team recording all agreements and areas of discussion. A trained research team member recorded detailed notes documenting points of agreement, disagreement, and key insights. Maps were photographed and systematically analysed to identify critical gaps, bottlenecks, and key stakeholders for in-depth investigation.

Step 2: In-Depth Key Informant Interviews

Based on findings from the supply chain mapping, semi-structured key informant interviews (KIIs) were conducted with the 15 identified stakeholders. The network mapping findings directly informed the content and focus of the interview guides in a deliberate, sequential manner. Specifically, actors who received high influence ratings and identified bottleneck nodes during the mapping exercise informed the development of targeted probes within the interview guides. For example, the five-star influence rating assigned to manufacturers prompted specific probes in the manufacturer guide around payment systems and production constraints, while the identification of financial flow disruptions during mapping generated explicit probes on government payment delays across multiple stakeholder guides. Separate, contextually tailored interview guides were developed for each stakeholder category, informed by the comprehensive literature review on THR implementation challenges, consultation with nutrition and implementation science experts, and preliminary findings from the broader intervention trial.

Interviews were conducted in Hindi (the local language) by trained research staff. The data collection team was stratified by organisational level: two project scientists with extensive qualitative research and nutrition expertise conducted interviews with state- and district-level officials; project technical staff holding Master's degrees in nutrition science conducted interviews with Anganwadi Workers and block-level coordinators. This strategy ensured contextual appropriateness and rapport with diverse participant groups. Each interview lasted 20-40 minutes. All interviews were digitally audio-recorded following written informed consent; interviews were supplemented with detailed field notes documenting non-verbal communication, environmental context, and emerging themes requiring follow-up.

Data management and analysis

All interviews were transcribed verbatim in Hindi by trained transcribers and translated into English by bilingual qualitative researchers familiar with the local socio-cultural context. To ensure translation accuracy, 20% of transcripts were back-translated and cross-verified. Data were analysed using thematic analysis following Braun and Clarke's framework [9], combining deductive codes with inductive codes emerging from the data. Coding was performed manually by two independent researchers, who reviewed transcripts line by line to identify key ideas and concepts. Independent coding enhanced objectivity and minimised individual bias.

Codes were subsequently organised into a hierarchical framework aligned with the study objectives, covering three major domains: operational challenges (procurement, storage, logistics), governance barriers (policy clarity, coordination, accountability), and human resource constraints (training, motivation, capacity). The codebook was developed iteratively: beginning with a deductive framework derived from the three study domains and expanded inductively as new codes emerged from the first three transcripts, which were independently coded by both researchers before the full codebook was finalised. A comprehensive codebook was developed to maintain consistency across analyses. The research team held bi-weekly meetings to review coding discrepancies, refine categories, and ensure analytical rigour through consensus. In instances of persistent coding disagreement, the principal investigator reviewed the contested codes as a third reviewer and provided a deciding interpretation. During qualitative analysis, emergent themes were synthesised into coherent narratives that illustrated variations across stakeholder groups, such as differences in perspectives between frontline workers and district officials.

For the integration of Net-Map and thematic analysis, interview narratives were cross-referenced with network influence scores during the analytical phase. For example, the five-star rating assigned to manufacturers during mapping was corroborated by interview accounts describing how payment delays to manufacturers cascaded disruptions across the entire supply system. One notable discrepancy observed between methods was that the District Program Officer received a moderate influence rating (three stars) during network mapping, yet interview accounts from AWWs and CDPOs suggested that DPO-level responsiveness to field-level complaints was perceived as lower still in practice, pointing to a gap between formal positional influence and practical operational responsiveness. 

Ethical considerations

Ethical approval was obtained from the Institute Human Ethical Committee, All India Institute of Medical Sciences (AIIMS) Bhopal (approval number: IHEC-LOP/2024/P24/044). The data collection team obtained written informed consent from all participants prior to data collection. The study maintained participant confidentiality through anonymisation; all transcripts and recordings were identified by participant codes rather than names and stored on password-protected, encrypted drives. Participants retained the right to refuse or withdraw from the study at any time without consequence.

## Results

Stakeholder characteristics

This study captured perspectives from the complete implementation hierarchy, from policy-making at the state level to service delivery at the grassroots. A total of 15 stakeholders participated in this qualitative analysis across different implementation levels of the THR program under ICDS. Table 1 presents the detailed characteristics of participants, including their roles, educational backgrounds, and years of experience in the program. AWWs represented diverse educational backgrounds, with many having completed only primary education, highlighting capacity-building needs. Administrative officials brought substantial program experience, while development partners provided technical expertise and strategic oversight perspectives. 

**Table 1:** Characteristics of study participants (N=15) THR = Take-Home Ration; AWC = Aangan Wadi Center; UNICEF = United Nations Children's Fund.

Stakeholder Category	Role/Position	Number (n)	Educational Background	Years of Experience	Location/Level
Frontline Workers	Anganwadi Workers (AWWs)	8	5th standard to Higher Secondary	2-15 years	Rural AWCs across 6 districts
Administrative Officials	Child Development Project Officers (CDPOs)	2	Graduate/Post-graduate	5-12 years	Block level
	District Program Officer (DPO)	1	Post-graduate	8 years	District level
	State Program Officer (SPO)	1	Post-graduate	10+ years	State level
Supply Chain	THR Manufacturing Manager	1	Graduate in Management	5 years	Production facility
Development Partners	UNICEF Representative	1	Technical specialist	7 years	State/National level
	Nutrition International (NI)	1	Program officer	6 years	National level

Network Mapping of Take-Home Ration Supply Chain

Net-mapping sessions were conducted to delineate the supply chain architecture of the THR program and assess institutional roles, influence levels, and resource flows among key actors. Participants from state, divisional, district, block, and community levels collaboratively developed the network map using colour-coded arrows to represent information (blue), financial (red), and food commodity (green) flows. Relative influence was rated on a five-star scale based on each actor's contribution to ensuring THR quality, timeliness, fund transfer efficiency, and adaptive management, as shown in Table 2 and Figure 1.

**Table 2:** Institutional influence ratings, functional roles, and resource flow dynamics in the THR supply chain network ★ Influence rated on a 1–5 scale (1 = low, 5 = high) through participatory net-mapping. RDA = Recommended Dietary Allowance; THR = Take-Home Ration; AWC = Anganwadi Centre; GOI = Government of India; QA = Quality Assurance; API = Application Programming Interface.

Actor	Influence	Key Responsibilities	Flows Out	Flows In
GOI Secretary	★★★	Issue guidelines; approve norms & APIs; oversee compliance	Information, Funds (50%), food items (Raw Materials)	Demand data, compliance reports
State and State Nutrition Committee	★★★★★	Set nutrient RDA values; finalise THR recipes; generate state demand	Information, Funds (50%), food standards	Implementation reports
Division/Manufacturers/Vendors	★★★★★	Procure raw materials; produce THR with QA; transport to districts	THR, quality reports, invoices	Raw material, funds
District Program Officer	★★★	Monitor distribution; compile state bills; authorise transport payments	Funds, transport data	THR receipts, billing documents, and Funds
Block Level Authorities	★★★★	Prepare distribution routes; verify and store THR; ensure timely delivery	THR Lab testing, transport logs	THR, funds
Anganwadi Centre (AWC)	★★★★★	Generate local demand; distribute THR; update Poshan Tracker	Beneficiary data; distribution logs	THR; guidelines and training material

**Figure 1:** Network map of the THR supply chain showing hierarchical actors, influence levels, and interconnected resource flows THR = Take-Home Ration. Colour codes: Blue = information flow; Red = financial flow; Green = food flow. Image Credit: This figure was created by the authors using Canva. The network structure was initially hand-drawn separately for district- and state-level systems and subsequently digitised and integrated into a single composite figure.

Six primary institutional actors were identified: The Government of India (GOI) Secretary, the State and State Nutrition Committee, the Division/Manufacturers/Vendors, the District Program Officer, the Block-Level Authorities, and the Anganwadi centres (AWCs). Three of these, the State Nutrition Committee, Division/Manufacturers/Vendors, and AWCs, received the maximum five-star rating, indicating their pivotal, non-substitutable roles within the THR supply chain. 

Backbone Actors and Hierarchical Dynamics

The THR supply chain operates through a vertically integrated yet interdependent hierarchy. Three actors form its operational backbone: the State Nutrition Committee, Division/Manufacturers/Vendors, and Anganwadi centres (AWCs), each translating national policy intent into tangible community benefit through distinct but complementary functions.

State nutrition committee (strategic policy hub): The State Nutrition Committee, comprising senior officials, AIIMS nutrition experts, and UNICEF advisors, functions as the central policy and coordination node. It establishes food standards through age- and group-specific Recommended Dietary Allowances (RDA), approves weekly THR recipes, and formulates cost-sharing ratios between central and state governments. The Committee consolidates district-level demand forecasts and communicates procurement targets directly to manufacturers. Upward flows of field feedback and implementation reports enable continuous program refinement. This dual-direction flow of information positions the Committee as the principal mechanism aligning national policy with state execution.

Division/manufacturers/vendors (commodity production and quality assurance): The manufacturing division operationalises state directives through procurement, production, and quality control. Raw materials (wheat, rice, soya) are acquired through closed-tender processes, ensuring quality and price stability. Multi-tiered quality assurance, including in-house and external laboratory testing, ensures product safety and compliance. Financial inflows from state accounts sustain production, while outflows include certified THR consignments, invoices, and quality reports. The manufacturer's role in converting policy prescriptions into standardised, consumable rations situates it as the operational core of the supply chain.

Anganwadi centers (frontline service and data nodes): AWCs represent the program's community interface, where policy outcomes manifest as household-level nutrition support. Through the Poshan Tracker digital platform, AWC workers register beneficiaries, generate localised demand, and record THR distribution. They verify consignments, maintain storage records, and collect beneficiary feedback on product use and acceptability. These real-time data streams support demand forecasting and inform upstream recipe or operational modifications. The AWC's proximity to communities and its dual role in service delivery and data generation confer both formal and informal influence within the system.

Intermediate Coordination and Oversight Actors

Block-Level Authorities coordinate logistics between districts and AWCs. Their responsibilities include route scheduling, receipt verification, storage management, and reimbursement of transport costs. Their four-star influence reflects substantial operational control within the distribution tier. District Program Officers provide fiscal oversight and program monitoring. They compile bills, authorise fund transfers, and review implementation reports from blocks and AWCs. Their role is supervisory rather than operational, resulting in moderate influence. GOI Secretary provides overarching policy direction and national monitoring. This role involves issuing Supplementary Nutrition Program guidelines, approving cost-sharing ratios, and reviewing compliance data from states.

Resource Flows and System Integration

Three interlinked flows sustain the THR system: Information flows (blue) connect all levels, translating policy downward and transmitting demand and feedback upward. These loops enable adaptive management and evidence-based decision-making. Financial flows (red) originate from state treasuries to fund production, transport, and AWC-level operations. Timely disbursement is essential to avoid production or distribution delays. Food commodity flows (green) trace the physical journey of THR from raw material procurement to manufacturing, warehousing, block distribution, and ultimately community-level consumption. Together, these flows create a vertically integrated but tightly coupled system whose resilience depends on synchronisation across nodes, as shown in Figure 1.

Key findings from multi-stakeholder perspectives on THR implementation challenges

Thematic analysis identified six overarching themes encompassing supply-side and demand-side dimensions of take-home ration (THR) implementation challenges. These themes encapsulated distinct but interconnected barriers across the program ecosystem: structural supply chain inefficiencies, product-community fit challenges, governance coordination gaps, workforce capacity deficits, community engagement limitations, and actionable stakeholder recommendations. Each theme contained between two and four sub-themes, capturing the nuanced perspectives of different stakeholder groups. Below, we present the major findings organised by theme, with illustrative quotes from representative participants. Supply chain complexity and governance gaps were the most cross-cutting themes, raised consistently by participants across all seven stakeholder levels. Product-community fit challenges were most prominently highlighted by AWWs and the THR manufacturer. Community engagement and SBCC barriers were predominantly surfaced by AWWs and development partners. While formal frequency counts are not presented consistent with Braun and Clarke's reflexive thematic analysis framework, which prioritises depth of interpretation over quantification, the differential salience of themes across stakeholder groups is noted to assist readers in contextualising the findings. Although some themes share conceptual territory (for example, governance gaps and community engagement limitations both reflect institutional fragmentation at different levels), they were maintained as distinct themes because they address qualitatively different aspects of the program ecosystem: one at the inter-departmental governance level and the other at the community-facing service delivery level, as shown in Table 3.

**Table 3:** Major themes, sub-themes, and illustrative verbatims from stakeholder interviews AWW = Anganwadi Worker; CDPO = Child Development Project Officer; AMB = Anaemia Mukt Bharat; IYCF = Infant and Young Child Feeding. Verbatim quotes from key informant interviews are anonymised; Block and Village numbers indicate study locations.

Major Theme	Sub-themes	Representative Verbatims
1. Supply Chain Complexity and Operational Barriers	1.1 Multi-level Supply Chain Structure	"Our process starts from Samuh with the board of directors from three districts... orders come from the women's office to the head office, then to the manufacturing plant" - Manufacturing Manager.
	1.2 Financial and Payment Challenges	"The biggest challenge is like milk powder or chana dal. They ask for the money first. Right now we have 3-4 crores in the plant," - Manufacturing Manager.
	1.3 Quality Control and Storage Issues	"Sometimes, sand is found in the Balahar packet. Then families refuse to eat it" - AWW, Village 2, Block 2
2. Product Acceptance and Utilisation Patterns	2.1 Taste and Sensory Acceptance	"Khichdi smells bad after storage, especially due to excess oil... Khichdi tastes bitter" - AWW, Village 4, Block 2
	2.2 Household Consumption Dynamics	Families roast halwa mix and make laddoos or barfi. But many use it for the whole family" - AWW, Village 1, Block 1
	2.3 Preparation Methods and Recipe Guidance	"It is written on the pouch, either you can inhale it directly in hot water, or you can heat it in milk" - Manufacturing Manager
3. Systemic Coordination and Governance Gaps	3.1 Inter-departmental Coordination	"Everyone has their own target... own system... own instruction" - State Program Officer
	3.2 Supervision and Monitoring Systems	"The supervisor comes once every 2–3 months. CDPO comes maybe once in 5–6 months" - AWW, Village 4, Block 1
	3.3 Technology Integration Challenges	"Face capture delays discourage beneficiaries; Jio network does not work well here" - AWW, Village 3, Block 2
4. Capacity Building and Human Resource Constraints	4.1 Training Gaps and Educational Barriers	"Many of us are 5th pass... we need basic, practical training regularly" - AWW, Village 1, Block 1
	4.2 Infrastructure and Resource Deficits	"Anganwadi has not been constructed; we operate from the school kitchen" - AWW, Village 2, Block 2
5. Community Engagement and SBCC	5.1 Communication Strategies and Tools	"We developed AMB flip book... with anaemia, fortification, IYCF" – Developmental Partner
	5.2 Language and Cultural Barriers	"They do not understand what we say... they speak in Malwa, in Bundel" --Block Administrative Official Block 1
	5.3 Community Resistance and Engagement	"Families say, 'What do you get? We have work to do.' But we still sit and talk" -AWW Village 2, Block 2
6. Stakeholder-Specific Recommendations	6.1 Supply Chain Improvements	"If Mahila Bal Vikas will give us some advance money... then we will get some things for making or supplying" - Manufacturing Manager
	6.2 Program Design Enhancements	"Separate packets for pregnant women and children will help avoid misuse" -AWW Village 2, Block 1
	6.3 Community-Level Interventions	"Sugar, oil should not be premixed—it spoils taste" -AWW Village 4, Block 1

Supply chain complexity and operational barriers

The take-home ration supply chain operates through a multi-layered administrative structure spanning state procurement offices, district aggregation facilities, block-level distribution hubs, and frontline Anganwadi centres. This hierarchical distribution pathway, while designed for centralised oversight and standardisation, generated recurrent operational bottlenecks at manufacturing, transport, and distribution stages. Three interconnected sub-themes characterise these supply-side barriers.

Multi-Level Supply Chain Structure and Distribution Flow Challenges

The THR distribution pathway involves multiple administrative tiers with distinct approval procedures and handoff points. A THR manufacturing manager described the operational process: "Our process starts from Samuh with the board of directors from three districts (Harda, Betul, Narmadapuram). Orders come from the Mahila Bal Vikas office in Bhopal and then to our manufacturing plant".

Each handoff across administrative levels introduced cumulative processing delays before products reached end-distribution points. Last-mile vulnerabilities further compromised product integrity during transit and unloading. The extended timeline from order placement to final delivery undermined responsiveness to supply fluctuations and created persistent inventory management challenges. Communication gaps between state procurement offices and block-level distribution hubs resulted in forecasting mismatches where demand signals did not align with supply availability, forcing redistribution from centres with surplus stock to those experiencing shortages. This reactive rather than proactive supply management pattern created cyclical availability gaps.

Financial and Payment System Bottlenecks

Government payment delays and deferred financing emerged as critical constraints limiting manufacturing capacity and production continuity. Manufacturers reported substantial pending receivables from the government that restricted their ability to procure raw materials from suppliers who demanded upfront payment. A THR manufacturing manager explained: "Suppliers demand payment upfront. We currently have ₹3-4 crore tied up in pending payments from the government".

These extended payment cycles, spanning multiple months between product delivery and government remittance, placed manufacturers under capital constraints that either disrupted production schedules or forced them to absorb costs through retained earnings, reducing their operational flexibility. The systemic mismatch between government fund availability and raw material procurement windows meant that even when funds were eventually disbursed, the opportunity to purchase raw materials at optimal market prices had often passed.

Quality Control Procedures and Storage Limitations

Quality assurance mechanisms existed at production facilities, including in-house testing of nutritional parameters and external verification through NABL-accredited laboratories. However, restricted storage capacity at manufacturing sites forced just-in-time procurement operations where manufacturers could maintain minimal buffer stocks. A THR manufacturing manager noted: "We cannot store more than 20-25 tonnes of any raw material. When supplies run out, we immediately issue a new purchase order".

This storage constraint reduced system resilience to supply disruptions and left the program vulnerable to raw material shortages that could interrupt production. At distribution endpoints, quality assurance failures undermined community acceptance. Contamination during transit, particularly sand in fortified premixes, prompted families to reject rations, directly reducing program effectiveness. Infrastructure inadequacies at service delivery sites compounded these quality concerns, where Anganwadi centres lacked secure storage facilities with appropriate climate control, exposing THR stocks to moisture, pests, and temperature fluctuations that degraded product quality before consumption.

Product acceptance and utilisation patterns

Community acceptance and household utilisation of take-home ration products exhibited substantial variation driven by sensory characteristics, preparation requirements, availability of time and resources, and household consumption dynamics. These demand-side factors directly determined whether target beneficiaries actually consumed prescribed rations and whether nutritional intake reached intended levels.

Taste Preferences and Sensory Acceptance Issues

Sensory characteristics, such as taste, post-storage odour, and texture, strongly influenced consumer acceptance of THR products and repeat consumption patterns. Multiple THR items were reported to develop off-flavours after storage, with khichdi-based products perceived as bitter, and rancid odours attributed to oil oxidation during extended storage periods. An Anganwadi worker (AWW Village 4, Block 2) described: "Khichdi smells bad after storage, especially due to excess oil. Khichdi tastes bitter".

This sensory degradation reflected a fundamental tension in product formulation: ingredients necessary for nutritional fortification (particularly soya protein to enhance amino acid profiles) contributed to unpalatable sensory profiles, reducing consumption despite improved nutritional adequacy. Monotonous daily consumption of identical products further reduced appeal and adherence. Communities preferred product variety, yet increasing formulation diversity required manufacturers to develop, test, and obtain approval for multiple products, a resource-intensive process with delayed regulatory timelines. The design dilemma persisted; stronger fortification improved nutritional value but compromised sensory acceptance, while taste-optimised formulations risked reducing nutritional density and program effectiveness.

Household Consumption Dynamics and Target-Group Sharing

Rations designated for specific vulnerable groups, children, pregnant women, and lactating mothers, were routinely shared across entire households rather than consumed by intended beneficiaries. An Anganwadi worker (AWW Village 3, Block 2) reported: Families roast halwa mix and make laddoos or barfi. But many use it for the whole family".

This intra-household sharing behaviour reflected rational household decision-making within contexts of food scarcity and cultural norms of equitable kinship-based food distribution. From program perspectives, sharing diluted the intended nutritional dose to individual vulnerable members, reducing targeting efficiency. However, from a household perspective, focusing on nutrition for a single household member while others remained undernourished conflicted with household food security strategies and social obligations. Working mothers faced additional utilisation constraints, as time requirements for daily preparation conflicted with their livelihood activities. Women engaged in agricultural or daily wage labour lacked consistent opportunity for daily THR preparation, leading them to prepare larger quantities less frequently, which inadvertently encouraged whole-household sharing rather than individual targeted consumption.

Preparation Methods and Recipe Guidance Limitations

Packaging provided only minimal and generic preparation instructions, limiting adaptation to local cooking practices, available fuel sources, and household preferences. Frontline workers routinely employed locally appropriate modifications, enriching khichdi with peanuts or ghee and adjusting cooking methods to available equipment, yet these practical adaptations were neither documented on packaging nor standardised across delivery points. A THR manufacturing manager confirmed: "The pouch instructions only state mixing with hot water or milk. No local recipes are provided".

This gap between standardised product design and contextual preparation realities constrained product acceptability and consistent nutrient delivery. The absence of localised recipe guidance was a missed opportunity to leverage frontline workers' knowledge and community preferences to enhance product utilisation. Communities lacked confidence to modify preparation methods despite possessing traditional knowledge of complementary ingredients and cooking techniques that could enhance both palatability and nutritional bioavailability.

Systemic coordination and governance gaps

The take-home ration program was implemented across multiple government departments with distinct reporting structures, targets, and operational instructions. This institutional fragmentation created governance challenges affecting program coherence, information flow, and adaptive management capacity.

Inter-Departmental Coordination Challenges and Structural Silos

Implementation responsibilities were distributed across departments, with unclear accountability and distinct performance metrics. A state program officer described: "Everyone has their own target, their own system, their own instruction". This departmental fragmentation generated redundant data collection systems, conflicting operational priorities, and inconsistent messaging to beneficiaries and implementation staff. However, positive collaboration examples existed at the local level, where Anganwadi workers, Auxiliary Nurse Midwives, and Accredited Social Health Activists worked as integrated teams on reproductive health and child survival initiatives. These instances of effective cross-sectoral cooperation demonstrated that collaboration was operationally feasible, yet such practices remained ad hoc and dependent on individual initiative rather than embedded within formal program structure. The absence of systemised coordination mechanisms prevented scalable replication of successful collaborative models.

Supervision and Monitoring System Effectiveness

Supervisory capacity was severely inadequate relative to program scale. An Anganwadi worker (AWW Village 1, Block 1) reported: "The supervisor comes once in two to three months. CDPO comes maybe once in five to six months". With approximately 97,000 anganwadi centres across the state, this supervisory visit frequency was insufficient for real-time troubleshooting, performance feedback, or adaptive program management. Digital monitoring tools partially compensated for in-person supervision limitations through the Poshan and Sampark apps, which achieved coverage of 70-80% of centres where internet connectivity permitted. However, unreliable connectivity in remote areas and inconsistent staff training on app functionality limited digital platform uptake precisely where alternative supervision mechanisms were weakest. This created accountability gaps, with the most geographically remote and potentially underserved populations receiving the least supervisory oversight and support.

Technology Integration Challenges and Digital System Barriers

Digital monitoring systems faced substantial operational hurdles that reduced functionality and user adoption. An Anganwadi worker (AWW Village 3, Block 1) noted: "Face capture delays discourage beneficiaries; Jio network is unreliable here". Poor network coverage, latency in biometric authentication features, and inadequate user training led to partial or inconsistent platform utilisation. Staff training on app updates was frequently inadequate, with workers uncertain about evolving platform functionality. These technical barriers impeded efficient data reporting and demotivated staff engagement with digital systems. The digital divide created by unequal internet access paradoxically disadvantaged remote populations who simultaneously faced the weakest traditional supervision mechanisms, concentrating program oversight challenges in the most difficult-to-serve geographies.

Capacity building and human resource constraints

Frontline workforce capacity emerged as a critical implementation bottleneck. Anganwadi workers, who serve as the primary interface between the program and communities, faced educational and training deficits that constrained service quality and program effectiveness.

Training Gaps and Educational Limitations Among Frontline Workers

Educational attainment among Anganwadi workers varied substantially, with many possessing only primary-level formal education. An Anganwadi worker (AWW Village 4, Block 2) reflected: "Many of us are 5th pass. We need basic, practical training regularly". Workers consistently requested recurrent, hands-on skill development opportunities focused on nutrition counselling, anthropometric measurement, and THR preparation techniques, ideally two to three times annually, to build and maintain competence. Program administrators acknowledged chronic underinvestment in training budgets, with funding for in-person skill development absent for extended periods. This training deficit directly limited the quality of community-facing services, constrained workers' ability to provide tailored guidance on product utilisation and dietary behaviour change, and reduced their confidence in program messaging. Specific skill gaps, including anthropometric assessment procedures and contextualised THR recipe preparation, remained unaddressed despite being identified as essential for effective program delivery.

Infrastructure and Resource Deficits Affecting Service Delivery

Physical infrastructure at many Anganwadi centres fell substantially short of program requirements. An Anganwadi worker (AWW Village 1, Block 2) reported: "Our Anganwadi has not been constructed. We operate from the school kitchen". Many centres operated from temporary or shared premises without dedicated space, adequate climate control, or secure storage facilities. The absence of dedicated THR storage exposed ration stocks to moisture, pests, and temperature fluctuations, creating food safety risks that could undermine community trust. The lack of child development materials and basic equipment reduced centres' appeal as community gathering spaces and constrained their capacity to deliver comprehensive early childhood development services. These infrastructure deficits, compounded by limited resource allocations for maintenance and supplies, created barriers to service quality that persisted independent of worker effort or commitment, representing structural rather than individual implementation challenges.

Community engagement and social behaviour change communication

Community mobilisation and behaviour change communication (SBCC) initiatives employed diverse strategies and communication channels, though their reach and cultural appropriateness varied substantially across urban and rural contexts and socioeconomic groups.

Communication Strategies and Tool Diversity Across Implementation Levels

Behaviour change communication initiatives deployed multiple delivery channels, flipbooks, radio jingles, short videos, and household counselling, reflecting pragmatic attempts to accommodate varied community access patterns and communication preferences. A development partner (an NGO program officer) representative explained: "We developed an anaemia-fortification flipbook and radio jingles to raise awareness among people in the easiest possible way".

However, digital channel effectiveness was highly context-dependent. Urban and peri-urban populations with access to smartphones, television, and internet connectivity could engage with YouTube-based content and WhatsApp-facilitated messaging. Rural populations with limited digital infrastructure found these channels inaccessible, creating unequal program exposure across geographic and socioeconomic strata. This fragmented channel approach, while reflecting adaptation to local infrastructure realities, risked reinforcing existing health communication inequities, with advantaged populations receiving digitally enhanced messaging while disadvantaged populations remained underexposed to behaviour change interventions.

Language and Cultural Adaptation Challenges

Standardised behaviour change materials frequently employed state-level languages that diverged substantially from local community dialects, creating comprehension gaps between program messaging and community understanding. A CDPO (Block Administrative Official Block 1) noted: "Beneficiaries often do not understand standard Hindi. They speak in Malwa, in Bundeli". This language misalignment represented a significant barrier to the effectiveness of behaviour change and contributed to perceived program irrelevance among communities. Conversely, frontline workers who communicated in local dialects and employed culturally grounded messaging examples achieved substantially better community receptiveness and engagement. The mismatch between standardised institutional materials and local communication contexts remained inadequately addressed despite frontline evidence that linguistic and cultural localisation substantially improved intervention effectiveness and community trust.

Community Resistance and Engagement Dynamics

Opportunity costs substantially limited household participation in program activities, particularly among economically vulnerable populations. An Anganwadi worker (AWW Village 2, Block 1) reported: "Labourers skip Village Health Nutrition Day (VHND) to avoid losing ₹300-₹350 daily wages". Daily wage losses deterred participation among labour-dependent households, reducing program exposure precisely among the most nutritionally vulnerable populations. This economic barrier reflected competing demands for immediate survival income and access to health services, rather than structural constraints or community indifference. Frontline workers employed adaptive engagement strategies, including brief, targeted household visits during non-work hours, to compensate for barriers to formal participation partially. These adaptive practices reflected both program commitment and recognition of structural constraints, though they necessarily reduced the comprehensiveness of behaviour change exposure compared to formal group sessions.

Stakeholder-specific implementation recommendations

Participants across all stakeholder groups, including manufacturing managers, Anganwadi workers, block and district administrators, and program officers, offered operationally grounded improvement suggestions reflecting their direct implementation experience and frontline knowledge of program operations.

Supply Chain and Production Enhancement Strategies

Manufacturing stakeholders proposed targeted interventions addressing identified financial and logistical constraints. A THR manufacturer recommended: "If Mahila Bal Vikas gives us some advance money, then we will get some things for making or supplying". Partial advance payments to manufacturers, contingent on production capacity and past performance, were proposed as mechanisms to stabilise raw material procurement and reduce production interruptions caused by delayed government remittance. Enhanced secondary packaging specifications were suggested to reduce contamination and breakage during distribution. Expedited approval pathways for product recipe modifications were recommended to increase manufacturer responsiveness to field-derived feedback on product acceptance and community preferences. These recommendations reflected recognition that supply chain reliability and product responsiveness required systemic support beyond individual manufacturer capacity.

Program Design and Service Delivery Improvements

Administrative stakeholders recommended systemic modifications to strengthen workforce quality and digital infrastructure. Merit-based recruitment coupled with competency assessment of Anganwadi workers was proposed as a mechanism to improve frontline service quality and program delivery consistency. Upgrading digital infrastructure at fair-price shops and distribution points was recommended to strengthen THR inventory tracking and reduce stock discrepancies. Product diversification, introducing varied THR flavours and formats, was suggested to reduce monotony and enhance acceptability across different population segments. Incorporating short, locally tailored video messages into behaviour change efforts was proposed as a strategy to leverage digital channels while maintaining cultural and linguistic relevance through community-based production.

Community-Level Operational Refinements

Frontline workers offered practical suggestions grounded in direct household engagement and implementation experience. An Anganwadi worker (AWW Village 4, Block 1) recommended: "Separate packets for pregnant women and children will help avoid misuse". Packaging modifications, particularly separate sachets designated for children and pregnant women, were suggested to facilitate targeted distribution and reduce intra-household sharing while acknowledging household decision-making autonomy. Component separation (maintaining sugar and oil as distinct ingredients rather than premixing) was recommended to allow households flexibility in product preparation, enabling taste adjustments and preserving palatability during storage. These community-derived suggestions reflected a sophisticated understanding of household consumption dynamics and represented low-cost, implementable modifications to enhance both targeting efficiency and product utilisation.

## Discussion

This multi-stakeholder qualitative analysis reveals the intertwined supply, demand, and governance obstacles that persistently weaken take-home ration (THR) program implementation under India's Integrated Child Development Services (ICDS). Using network mapping, this study reveals that the State Nutrition Committee, manufacturers, and Anganwadi centres are linchpins of program success, their central roles conferring both authority and responsibility. However, this concentrated influence produces systemic vulnerabilities when these backbone actors experience disruptions; the consequences quickly ripple through all layers of the system, highlighting how single points of failure fundamentally threaten program continuity.

This study examined implementation barriers from stakeholder perspectives and did not directly measure nutritional outcomes such as stunting, wasting, or program utilization rates. Any associations between the identified supply-side barriers and child nutritional outcomes referenced in this discussion are inferred from the existing literature and should not be interpreted as empirically established causal relationships within this study's design. Conclusions are appropriately framed as stakeholder-derived, context-specific insights rather than system-wide definitive findings.

These results not only reaffirm concerns seen in earlier evaluations, including chronic supply chain breakdowns, quality assurance shortfalls, and limited frontline workforce capacity, but also deepen understanding of how these issues emerge from the program's structural design. For example, prior evidence from Maharashtra highlighted contamination in ration packets, poor storage conditions, and limited community awareness [10]. Similar investigations in Rajasthan and Jharkhand reported acute ration stockouts linked to supplier payment delays, findings that align closely with financial constraints and implementation lags observed by manufacturers in this study's setting [11]. Rather than reflecting isolated incidents, such patterns surface across diverse geographies and stakeholders, suggesting these are foundational weaknesses in program architecture rather than exceptions.

The hierarchical structure in the network mapping is not inherently problematic; centralisation can bring oversight and efficiency. However, a lack of redundancy or adaptable feedback mechanisms can hinder resilience and adaptation, compounding the system's fragility. For instance, as documented here and in evaluations employing participatory network approaches, essential communication and resource flows often move in parallel silos, distanced from the ground realities and needs uniquely understood by frontline staff [12]. Without formalised channels to convey practical feedback on product use and household realities upward, frontline actors remain unable to influence significant aspects of program design, such as recipe alterations or packaging changes, irrespective of their acute awareness of what works locally [13].

Similarly, while multi-tiered administrative supply chains are intended to reinforce quality and accountability, they often introduce cumulative logistical delays, poorly managed inventories, and stifled responsiveness at the local level. Evidence from comparable nutritional interventions in Bangladesh, for instance, shows that buffer stocks, decentralised supply chain management, and prompt procurement approvals directly improve system resilience and availability [14]. The large-scale payment delays reported by Indian manufacturers, as echoed in public sector procurement research, significantly dampen suppliers' flexibility, forcing them either to curtail production or to rely on reserves, both of which ultimately risk stockouts and program interruptions [15]. This financial-logistical misalignment created inefficiencies that cascaded through the production system, preventing consistent ration availability at distribution endpoints.

Quality assurance, critical for both safety and community trust, continues to be undermined by field-level challenges [16]. Although production facilities maintain robust nutritional and laboratory verification, the realities of rural transport and insufficient local infrastructure expose products to unacceptable risks of moisture, temperature swings, and pest contamination. Anganwadi workers reports of contamination, such as finding sand in rations, highlight the practical disconnect between formal quality protocols and everyday delivery. Studies from large-scale food fortification programs confirm that robust transport, infrastructure, and storage solutions are as important as technical quality control [17].

Another pivotal finding is the persistent disconnect between formulating optimally fortified products and achieving community acceptance. While the inclusion of soya protein and other nutrients is mandated for child health, these same ingredients frequently undermine product palatability, ultimately reducing uptake. Controlled trials and systematic reviews acknowledge that nutrient-fortified products do not always outperform unfortified options in acceptability, particularly when distributed under non-ideal field conditions that accentuate flavour and texture degradation over time. The underlying lesson is clear without engaging households in iterative product development and prioritising sensory considerations alongside nutritional value, intended health impacts may never be realised [18,19].

Intra-household ration sharing, a recurring observation in food-insecure settings, further complicates targeting. Culled from both this and broader studies, household rations intended for children or mothers are commonly shared among all family members, particularly when household food insecurity is high and social norms discourage selective allocation [20]. It raises sensible questions about the appropriateness of recipient-focused targeting models and supports consideration of more flexible, household-oriented approaches that align with local values while maximising nutritional benefits.

Preparation guidance also warrants rethinking. Uniform, generic instructions provided on packages are often disconnected from regional food cultures and household practices, missing clear opportunities to integrate frontline expertise and community foodways into program delivery. Research in both Indian and African contexts underscores that nutritional impact depends as much on cultural adaptability and practical utilisation as on the nutrient profile itself. In this study, Anganwadi workers routinely modified recipes to local tastes, but these innovations remain undocumented, limiting their broader adoption and missing a chance to standardise best practice [21].

Governance constraints, fragmented cross-sector coordination, sporadic supervision, and challenges with digital monitoring affect every level of service delivery. While the expansion of digital platforms has improved coverage in well-connected areas, both this analysis and global digital health reviews demonstrate that these gains are undermined by unreliable internet, inadequate training, and gaps in infrastructure, particularly in remote regions where oversight is needed most [22]. These same regions are often the least supervised due to logistical barriers, exacerbating inequities in program reach.

Workforce capacity stands as another crucial lever for impact. Anganwadi workers, often with primary education and little ongoing training, are asked to deliver increasingly technical interventions without the support or upskilling necessary for high-quality service provision. Global and Indian evidence strongly support investments in practical training, competency-based recruitment, and workforce expansion not only to improve service delivery but to foster motivation, social recognition, and retention [23].

Stakeholder-sourced recommendations, ranging from advance payments to manufacturers and improved packaging to diversified rations and merit-based worker recruitment, are both practical and grounded in lived experience. Critically, evidence from this study suggests that the identified barriers are structurally interdependent, and that isolated, single-component interventions may have limited impact without coordinated systems-level reform. Experience from participatory action research and health system strengthening globally affirms that, without meaningful routes for distributed knowledge to inform adaptive design, implementation will always lag behind aspiration [24].

Despite limitations of geographic and sample breadth and the inherent biases that come from close programmatic involvement, these findings offer a compelling, actionable set of priorities. Stabilising procurement by combining advance payments with robust payment systems, strengthening logistics and secondary packaging, investing in recurrent workforce training, supporting product diversification, and enhancing community engagement through locally adaptive communication and ingredient packaging all have immediate feasibility and apparent impact [25,26]. However, only coordinated pursuit of these reforms, rather than piecemeal or siloed efforts, will harness potential synergies and address the system’s interconnected weaknesses [27].

Future research should prioritise real-world, longitudinal assessments of reform impact; the integration of coverage and process data using mixed-methods; geographic expansion to illuminate universal versus context-specific challenges; participatory co-design approaches to fuel local innovation; and economic modelling to generate compelling investment cases. Ultimately, the preponderance of evidence, locally and globally, converges on a central lesson [28]: technical solutions are vital, but only transformative when they are unlocked by responsive governance, empowered frontlines, and a design ethos that truly values lived expertise as much as formal protocols.

Strengths and limitations

This qualitative study employs rigorous mixed-methods, combining network mapping and in-depth interviews across seven organisational tiers, capturing systemic interdependencies among supply, governance, and community engagement that are rarely documented in THR evaluations. Maximum variation purposive sampling of 15 stakeholders and independent dual coding enhance analytical credibility. The novel application of Net-Map methodology within the THR context represents a specific methodological contribution of this study: by visually and participatorily revealing structural vulnerabilities and non-substitutable backbone actors, Net-Map surfaced systemic interdependencies that conventional interview-only designs may not readily expose.

However, geographic restriction to the Hoshangabad district limits generalizability across Indian states with differing administrative structures. It is acknowledged that Hoshangabad district's administrative and infrastructural context may differ from states with substantially higher or lower NFHS-5 nutritional burden indicators, and findings should be interpreted within this geographic boundary. The cross-sectional design cannot capture seasonal variations in availability and storage degradation, while potential social desirability bias may influence government and manufacturer responses, given the research team's prior program involvement. The inability to directly observe implementation processes, rather than relying solely on stakeholder accounts, restricts triangulation with actual supply chain delays and quality failures.

The over-representation of Anganwadi Workers (n=8, 53%) means findings may disproportionately reflect frontline service delivery perspectives, with higher-level governance and fiscal viewpoints captured through only four administrative and development partner participants, who are less comprehensively represented. Future studies should deliberately oversample higher-level stakeholders to achieve a more balanced distribution. The study relied entirely on stakeholder self-reports and did not incorporate direct observational methods, document review (e.g., program monitoring reports, government payment records), or beneficiary-level validation. The absence of these triangulation sources means reported barriers could not be independently verified against programmatic records or beneficiary experiences. Member checking was not formally conducted; however, the research team's prolonged engagement with the study setting and the corroboration of findings across multiple stakeholder groups served as a partial compensatory mechanism for establishing confirmability. No quantitative frequency analysis of themes was undertaken, consistent with Braun and Clarke's reflexive thematic analysis framework; however, this means formal comparisons of theme prominence cannot be made. Nutritional outcomes were not directly measured within the design of this sub-study; however, these parameters are being assessed as part of the Nutritional Status Enhancement of Children through Behaviour Change Communication and Take-Home Ration (NECCTAR) trial, and associations between the identified barriers and child nutritional status are interpreted in that broader study context.

## Conclusions

This multi-stakeholder analysis demonstrates that the Take-Home Ration program's limited effectiveness arises from structural fragilities embedded within its supply chain and governance architecture. Excessive centralisation, fiscal bottlenecks, fragmented inter-departmental coordination, and chronic workforce deficits collectively erode accountability and operational reliability. Key nodes, the State Nutrition Committee, manufacturing units, and Anganwadi Centres, function as non-redundant actors whose interdependencies generate systemic vulnerability. Evidence from this study suggests that the identified barriers are structurally interdependent, and that isolated, single-component interventions may have limited impact without coordinated systems-level reform. Misalignment between product fortification standards and household sensory preferences further diminishes utilisation, while frontline innovations such as localised recipes, adaptive community engagement, and contextualised product modifications remain excluded from formal policy learning cycles. Advancing THR effectiveness requires a paradigmatic shift from hierarchical compliance to adaptive governance that institutionalises frontline knowledge. Priorities include fiscal predictability, decentralised decision-making, cross-sectoral coordination, and culturally responsive behaviour change communication. Embedding these reforms can strengthen supply chain resilience, enhance program acceptability, and accelerate sustainable reductions in childhood undernutrition across resource-constrained settings.

## Appendices

Note: The interview guides presented in the appendices are English-language working translations, that were developed and administered verbally in Hindi during data collection. Minor typographical and formatting inconsistencies in the appendices reflect the working nature of these translated documents and do not represent the form in which they were used in the field. 

Interview Guide -1

The Nutritional Status Enhancement of Children through Behaviour Change Communication and Take-Home Ration (NECCTAR) Trial

Interview Guide for AWC level functionaries (Anganwadi Worker, and Anganwadi Helper)

Objectives of the tool: (a) To understand various aspects of the program and it’s functioning in the community, (b) To understand the stakeholders’ perceptions regarding their needs, and challenges faced by them at various steps of the supply chain of the the program, and (c) To explore the key entry points of intervention at different stages of the supply chain to strengthen the program and diversify the foods/meals given under the program.Target participants: Anganwadi Worker and Anganwadi Helper introduction

Hello, I am ………………………………. from AIIMS, Bhopal. I am part of the NECCTAR trial research team exploring the current status of the THRs being provided in your community. We want to understand the take-home ration (THR) food supplied in your area like where the raw ingredients are obtained from, where and how manufactured and processed, and how these are supplied to the Anganwadis. We wish to know how these THR foods are distributed from the Anganwadis. We also want to know how the mothers and the community are informed and educated about nutrition and feeding of the children, including the THR foods. We wish to find out how the nutrition status of the children can be improved further and how the ICDS program can perform better. The purpose of this study is to improve the dietary practices for children, including the THR food use. The final goal is to reduce malnutrition in young children.

This is just a conversation, and there are no right or wrong answers. If you are okay, I will be writing notes and if you agree, I will also use this recorder for recording our conversation, so that I don't miss things. The interview will take around 30 minutes. Do you agree and consent to the interview?

1. Yes, 2. No

If consent is given by the participant, proceed with the interaction/interview.

1. Stakeholder information

**Table 4:** Stakeholder information

SN	Item	Response	SN	Item	Response
1.1	State		1.2	District	
1.3	Block		1.4	Sector area	
1.5	PHC SC		1.6	AWC Code	
1.7	AWC name		1.8	Village/Area name	
1.9	Respondent name		1.10	Designation	AWW AWH
1.11	Period of service	Years	1.12	Area Category	Rural Urban

2. Information about the nutrition services and Take-Home Ration (THR)

2.1.  May I request you to tell us about the production and supply of the Take Home Ration (THR) products or items to your AWC?

Probe: Production (place, who prepares, source of ingredients, production process, packaging), indent and supply (frequency, mode, and timeliness)

2.2.  May I request you to tell us about the distribution, acceptance, and utilization of the THR for the children in the households or your area? If used, why? If not used, why?

Probes: Distribution from AWC (frequency and amount), acceptance (perceived quality and benefit, sociocultural suitability), utilization (use for the children, mode of use-cooked or uncooked, use by other family members, use for other purposes), possible reasons for use and/or non-use. If the THR acceptance is reported as low, there is a need to explore why (like product quality, taste, apprehensions, cultural practices, cooking needs, or any other resistance). 

2.3. In your opinion, what are the challenges related to THR for use in children in your area? How can these challenges be addressed?

Probes: THR-related (quality, ingredients, preparation, packaging), supply and distribution (quantity, frequency, regularity, storage, wastage, distribution, procedural issues), use at households (acceptance, preparation, and cooking).

2.4. May I request you to tell us about the supervision, monitoring, and support you receive from the sector supervisor and CDPO for the service delivery? How can this be improved?

Probe: who supervises/monitors, schedule or frequency, activities done, quality, feedback, factors influencing, challenges, and potential improvements.

3. Information about the IYCF practices in the community

3.1. In your opinion, what are the usual practices related to complementary feeding for young children by the mothers/caretakers in this area?

Probe: Timing of initiation, types of food and food diversity, adequacy of food, sociocultural norms and practices, use of market baby foods and health drinks.

3.2. In your opinion, how do the mothers/caretakers/family members of children with undernutrition accept your advice and counseling? If they do not follow your counseling, why?

Probe: recognition of undernutrition status, acceptance and compliance to special foods for MAM and SAM, and anemia, possible reasons for acceptance or refusal, any sociocultural practices or influences.

4. Information about Social and Behaviour Change Communication (SBCC)

4.1. May I request you to tell us how you usually provide the nutrition and health education and/or counseling to the mothers/beneficiaries and community? 

Probes: types of activities, places (AWC or households or community meetings/groups); schedule, tools/job aids used (pictures/flip charts/audio-visuals/verbal); positioning of THR (need, importance, ingredients, quality) and home food. 

4.2. In your opinion, what are the challenges experienced by you related to nutrition and health education and counseling activities? What are the potential influencing factors? How could these challenges be addressed?

Probe: participant related (interest, time constraints, perceived benefit), content and channel (IEC/BCC content, local culture and language appropriateness, channel), positive influencers, negative influencers, possible modalities to address.

5. Information about community engagement, coordination, and accountability

5.1. May I request you to tell us about the participation of the health functionaries (ASHA, ANM, CHO and others) in your area in the nutrition and health education activities (including THR and management of undernutrition)?

Probes: how the health functionaries participate, relationships with AWW/AWH, opportunities or platforms (VHND, community meetings, nutrition checkup, healthcare).

5.2. May I request you to tell us about the support and contributions by other persons, groups, or organizations for the nutrition and health activities in your area? If yes, how?

Probe: who participates/contributes (community/panchayat/Jaanch Committee/ Mother’s Committee/NGO/SHG/CBO/teachers/other persons/organisation), mode of participation, schedule or frequency, challenges.

5.3. In your opinion, what are the challenges experienced related to community engagement and participation in nutrition and health education activities in your area? What are the potential influencing factors? How could these challenges be addressed?

Probe: challenges, positive influencers, negative influencers, reasons, person/group who could contribute, how?

6. Needs for improving the service delivery

6.1.  In your opinion, what can be done to assist the AWC team (or you) in improving the nutrition and health services and THR-related activities in your area? How can the THR acceptance and use for children be improved?

Probe: counselling or IEC/BCC/SBCC-related activities (communication skill, competence, confidence, provision of job aids, audiovisual materials), THR recipe and use related (preparation and use demonstration), undernutrition (nutritional assessment and management)

7. Closure

7.1.  Before closing the interaction, would you like to suggest anything that could improve the nutrition and health service delivery at the AWCs?

We thank you for your critical contribution.

Interview guide- 2

The NECCTAR Trial

Interview Guide for ICDS supervisory functionaries (ICDS Sector Supervisor and CDPO).

Objectives of the tool: (a) To understand various aspects of the program and it’s functioning in the community, (b) To understand the stakeholders’ perceptions regarding their needs, and challenges faced by them at various steps of the supply chain of the program, and (c) To explore the key entry points of intervention at different stages of the supply chain to strengthen the program and diversify the foods/meals given under the program.

Target group: ICDS Sector Supervisor and CDPO

Introduction:

Hello, I am ………………………………. from AIIMS, Bhopal. I am part of the NECCTAR trial research team exploring the current situation of the THRs being provided in your community. We want to understand the supply chain of the program by finding out where the raw ingredients are obtained from, the manufacturing and processing involved, distribution of the prepared THR to the Anganwadi Centres (AWCs), and final delivery to the beneficiaries. Along with this, we want to know if any communication strategies for nutrition education are being used in your community. We wish to find out ways of strengthening this program to improve the health and nutritional status of the community. The purpose is to strengthen and improve the program modalities leading to diversity in the diets of the beneficiaries and making them food secure. The final goal is to reduce malnutrition in young children.

This is just a conversation, and there are no right or wrong answers. If you are okay, I will be writing notes and if you agree, I will also use this recorder for recording our conversation, so that I don't miss things. The interview will take around 30 minutes. Do you agree and consent to the interview?

1. Yes, 2. No

If consent is given by the participant, proceed with the interaction/interview.

1. Stakeholder information

**Table 5:** Stakeholder information

SN	Item	Response	SN	Item	Response
1.1	State		1.2	District	
1.3	Block		1.4	Sector area	
1.5	Respondent name		1.6	Designation	
1.7	Period of service		1.8	Area category	Rural Urban

2. Information about the ICDS programme and the Take Home Ration (THR).

2.1. May I request you to tell us about the strategy and efforts under the ICDS program and Take Home Ration (THR) in the district?

Probe: enrollment of beneficiaries, coverage for nutrition services, any special financial package, special effort, THR products (ingredients, special adaptation/modification).

2.2. May I request you to tell us about the production and supply of the Take Home Ration (THR) products or items to the AWCs in your area?

Probe: Production (place, who prepares, source of ingredients, production process, packaging), indent and supply (frequency, mode, and timeliness).

2.3. May I request you to tell us about the distribution, acceptance and utilization of the THR for the children in the households of your area? If used, why? If not used, why?

Probes: Distribution from AWC (frequency, and amount), acceptance (perceived quality and benefit, sociocultural suitability), utilization (use for children, mode of use-cooked or uncooked, use by other family members, use for other purposes), possible reasons for use and/or not use.

2.4. In your opinion, what are the challenges related to THR for use in children in your area? How can these challenges be addressed?

Probes: THR related (quality, ingredients, preparation, packaging), supply and distribution (quantity, frequency, regularity, storage, wastage, distribution, procedural issues), use at households (acceptance, preparation and cooking).

2.5. May I request you to tell us how the formulation and ingredient composition for the THR are decided for the district?

Probe: who decides, factors considered, when last revision done, any special adaptation.

3. May I request you to tell us how the activities at the AWCs in your area are monitored and supervised? What are the challenges faced/experienced and how are these being addressed?

Probe: who supervises/monitors, schedule or frequency, activities done, quality, feedback, factors influence and challenges, modalities or efforts to address them. 

4. Information about the IYCF practices in the community

4.1. In your opinion, what are the usual practices related to complementary feeding for young children by the mothers/caretakers in this area?

Probe: onset of complementary feeding, adequacy of food, food diversity, sociocultural norms and practices.

4.2. In your opinion, how do the mothers/caretakers/family members of children with undernutrition accept the advice and counseling by the AWC team? If they do not follow your counseling, why? 

Probe: recognition of normal and undernutrition status, seeking assistance, acceptance and compliance to special foods for MAM and SAM, and anemia cases, possible reasons for acceptance or refusal, any sociocultural practices or influences.

5. Information about Social and Behaviour Change Communication (SBCC).

5.1. May I request you to tell us how the AWCs in the area provide nutrition and health education and counseling activities to the beneficiaries and community?

Probes: types of activities, places- AWC or households; participants, schedule, focus areas, tools/job aids used.

5.2. In your opinion, what are the challenges experienced by the AWCs in your area while delivering the nutrition and health education and counseling activities? What are the potential influencing factors? How could these challenges be addressed?

Probe participant related (interest, time constraints, perceived benefit), content and channel (IEC/BCC content, local culture and language appropriateness, channel), positive influencers, negative influencers, influence of social media and mass media, possible modalities to reach the community and address the issues.

6. Information about community engagement, coordination and accountability

6.1. May I request you to tell us about the participation of the health functionaries (ASHA, ANM, CHO and others) of your area and the district in the nutrition and health education activities (including THR and management of undernutrition)?

Probes: how health functionaries participate, relationships with AWW/AWH, opportunities or platforms (VHND, community meetings, nutrition checkup), referral and management of undernutrition.

6.2. May I request you to tell us about the support and contribution by other persons, groups, or organizations for the nutrition and health activities in your area? If yes, how?

Probe: who participate/contribute (community/panchayat/Jaanch Committee/ Mother’s Committee/ NGO/SHG/CBO/teachers/ others persons/organisation), mode of participation, schedule or frequency, challenges.

6.3. In your opinion, what are the challenges related to community engagement and participation in nutrition and health education activities in your area? What are the potential influencing factors? How could these challenges be addressed?

Probe: challenges, positive influencers, negative influencers, reasons, person/group who could contribute, how?

7. Needs for improving the service delivery.

7.1. In your opinion, what can be done to assist the AWC team (AWWs and AWHs) to improve the nutrition and health services and THR-related activities in your area?

Probe: counseling or IEC/BCC/SBCC related activities (communication skill, competence, confidence, provision of job aids, audiovisual materials), THR recipe and use related (preparation and use demonstration), undernutrition (nutritional assessment and management).

8. Closure

8.1. Before closing the interaction, would you like to suggest anything that could improve the THR services and coverage for children? Would you like to suggest anything to improve the nutrition and health service delivery at the AWCs?

We thank you for your critical contribution.

Interview guide-3

The NECCTAR Trial

Interview Guide for WCD Program Officer (District WCD Officer, State WCD Program Officer).

Objectives of the tool: (a) To understand various aspects of the program and its functioning in the community, (b) To understand the stakeholders’ perceptions regarding their needs and challenges faced by them at various steps of the supply chain of the program, (c) To explore the key entry points of intervention at different stages of the supply chain to strengthen the program and diversify the foods/meals given under the program.

Target group: District and State WCD Program Officer.

Introduction: 

Hello, I am ………………………………. from AIIMS, Bhopal. I am part of the NECCTAR trial research team exploring the current situation of the THRs being provided in your community. We want to understand the supply chain of the program by finding out where the raw ingredients are obtained from, the manufacturing and processing involved, the distribution of the prepared THR to the Anganwadi Centres (AWCs) and final delivery to the beneficiaries. Along with this, we want to know if any communication strategies for nutrition education are being used in your community. We wish to find out ways of strengthening this program to improve the health and nutritional status of the community. The purpose is to strengthen and improve the program modalities leading to diversity in the diets of the beneficiaries and making them food secure. The final goal is to reduce malnutrition in young children.

This is just a conversation, and there are no right or wrong answers. If you are okay, I will be writing notes, and if you agree, I will also use this recorder for recording our conversation, so that I don't miss things. The interview will take around 30 minutes. Do you agree and consent to the interview?

1. Yes, 2. No

If consent is given by the participant, proceed with the interaction/interview.

1. Stakeholder information

**Table 6:** Stakeholder information

SN	Item	Response	SN	Item	Response
1.1	State		1.2	District	
1.3	Respondent name		1.4	Designation	

2. General information about the ICDS programme and the Take Home Ration (THR).

2.1. May I request you to tell us about the special strategy and efforts targeted at child nutrition under the ICDS program in the state and/or the select district (study district name)?

Probe: enrollment of beneficiaries, coverage for nutrition services, any special financial package, special effort, any CSR activity, any community processes

2.2. May I request you to tell us about the strategy, decision-making, and guideline development for Take Home Ration (THR) products, preparation, and supply in the state and select district (study district name)?

Probe: products, composition, suitability for beneficiaries, any special adaptation/modification, manufacturer(s), source of raw materials, quality check and certification, packaging and labeling, supply

2.3.  In your opinion, how are the beneficiaries/households and community accepting and utilizing the THRs supplied under the ICDS program? What are the possible reasons?

Probes: acceptance (perceived quality and benefit, sociocultural suitability), utilization (use for children, use by other family members, use for other purposes), possible reasons for use and/or non-use.

2.4.  In your opinion, what are the challenges related to the THR production, procurement, supply, and acceptance by beneficiaries? How can these be addressed?

Probes: THR related (quality, ingredients, preparation, packaging), supply and distribution (quantity, frequency, regularity, storage, wastage), household acceptance and use

2.5.  May I request you to tell us how the activities at the AWCs in your area are monitored and supervised? What are the challenges faced/experienced, and how are these being addressed?

Probe: who supervises/monitors, schedule or frequency, activities done, quality, feedback, factors influencing and challenges, modalities or efforts to address them. 

3. Information about community and household IYCF practices.

3.1. In your opinion, what activities have been undertaken or efforts made to improve the household-level IYCF practices? What have been the experiences with such efforts?

Probe: efforts to improve complementary feeding, dietary diversity for children, challenges, and lessons

3.2. In your opinion, what are the challenges related to complementary feeding in young children? How could these be addressed? Who all can contribute?

Probe: challenges, person/group who could contribute, how?

4. Information about Social and Behaviour Change Communication (SBCC).

4.1. May I request you to tell us about the overall communication strategy and actions being adopted under the ICDS program related to the young child feeding and THR use?

Probe: any specific communication strategy, campaign, targeting nutrition, THR or any other, use of job aids/tools by the ICDS team at different levels.

4.2. In your opinion, what efforts have been made or are being made for capacity building of the AWC and/or ICDS teams in delivering the nutrition and health education activities? What are the potential influencing factors? How could these challenges be addressed?

Probe: AWC team’s competence and confidence, IEC/BCC/SBCC materials and/or tools/job aids (content, local culture and language appropriateness, channel), training methods, influencers (positive and negative), possible modalities to address.

5. Information about coordination, community engagement, and accountability

5.1. May I request you to tell us about the participation of the health functionaries and officials at different levels in the state and district for ICDS-related activities? What coordination mechanisms are in place?

Probes: roles played and contributions, coordination mechanisms and platforms, appropriateness, challenges and how addressed.  

5.2. May I request you to tell us about the support and contribution by other departments, persons, groups, or organizations for the nutrition and health activities in the state and select district? If yes, how?

Probe: who participate/contribute (community/panchayat/Jaanch Committee/ Mother’s Committee/ NGO/SHG/CBO/teachers/ other persons/organisation), mode of participation, schedule or frequency, challenges and how addressed.

5.3. In your opinion, what are the challenges experienced related to the community engagement and participation in ICDS services in the state and select district? What are the potential influencing factors? How could these challenges be addressed?

Probe: challenges, positive influencers, negative influencers, reasons, person/group who could contribute, how?

6. Closure

6.1. Before closing the interaction, would you like to suggest anything that could improve the nutrition and health service delivery by the ICDS team?

We thank you for your critical contribution.

Interview guide-4

The NECCTAR Trial

KII Guide for THR Manufacturer and Supply Agency.

Objectives of the tool: (a) To understand various aspects of the THR production and supply, (b) To understand the processes, needs, and challenges at various steps of the supply chain THR.

Target participant: THR manufacturer or THR Supply Agency.

Introduction

Hello, I am ………………………………. from  AIIMS Bhopal. I am part of the NECCTAR trial research team exploring the current status of the THRs being provided in your community. We want to understand the supply chain of the program by finding out where the raw ingredients are obtained from, the manufacturing and processing involved, the distribution of the prepared THR to the Anganwadi Centres (AWCs), and final delivery to the beneficiaries.

Your opinion is critical to improving the overall function of the program and utilization of the THR. This is just a conversation, and there are no right or wrong answers. If you are okay, I will be taking notes, and if you agree, I will also use this recorder for recording our conversation, so that I don't miss things. The interview will take around 30 minutes. Do you agree and consent to the interview?

1. Yes, 2. No

If consent is given by the participant, proceed with the interaction/interview.

1. Stakeholder information

**Table 7:** Stakeholder Information

SN	Item		SN	Item	
1.1	State		1.2	District	
1.3	Block		1.4	Name of agency	
1.5	Category of agency	Government agency Private agency SHG Other (specify)	1.6	Role of agency	Manufacturer Supplier Other
1.7	Location of agency		1.8	Supply area of the agency	Districts ……… Blocks …………
1.9	Respondent name		1.10	Designation/ Job description	

2. General information about the agency and products

2.1. May I request you to tell us about your agency/organization, its activities and the products manufactured/ handled/supplied?

Probe: type of organization, location, years of operation, activities undertaken, if SHG/NGO- membership strength, products manufactured or supplied, years of association with the ICDS and THR.

3. Take Home Ration (THR) products manufacturing and distribution

3.1. May I request you to tell us about the Take Home Ration (THR) foods and/or food products that are manufactured/supplied by your agency/organization? Who decides the composition and recipe, and how? Which areas are being supplied by your organization?

Probe: types of products, guidelines issued, place(s) of manufacturing, source of raw materials, process of procurement, manufacturing process, production amount/volume and schedule, packaging and labeling.

3.2. May I request you to tell us about the quality checks and testing done for the THR products manufactured or supplied by your agency?

Probe: quality check and testing, types of testing, components tested, laboratory, frequency, certification, shelf-life checking

3.3. May I request you to tell us about the process of indenting of raw ingredients, ordering, supply, logistics and distribution of THR from your unit to the AWCs?

Probe: forecasting, quantity, ordering, scheduling, frequency, procedural issues, storage, distribution,

3.4. May I request you to tell us about the challenges related to the THR production, packaging, testing, supply and logistics, experienced by you/ your agency?

Probes: challenges related to the administrative, raw material procurement, manufacturing, testing, packaging, labeling, distribution and supply, forecasting, payments, and others.

4. Take-Home Ration (THR) product usage

4.1. May I request you to tell us about the food recipes that are recommended and/or can be prepared using the THRs for feeding young children, and are there cookbooks documenting these?

Probe: types of recipes, cookbooks, who developed and printed, any updates done, availability, and distribution.

4.2. In your opinion, how is/are the THR products (manufactured/supplied by you/your agency) being utilized by the families/households? What are the possible reasons?

Probes: acceptance of the THR, mode of use, use for the child, use for other purposes, perceived quality and benefit, sociocultural compatibility.

4.3. In your opinion, how can the THR products be further improved or modified to make it more acceptable and used by the mothers and households?

Probe: use of local ingredients, composition, manufacturing process, packaging, quality checking, transportation, storage, reducing wastage, preparation/cooking needs, recipes

5. Closure

5.1. Before closing the interaction, would you like to suggest anything that could improve the nutrition service delivery by the ICDS team and improve the nutritional status of children?

We thank you for your critical contribution.

Interview guide-5

The NECCTAR Trial

Interview Guide for Partners-State and District Level (UNICEF, State Mother NGO, District NGO).

Objectives of the tool: (a) To understand various aspects of the program and its functioning in the community, (b) To understand the stakeholders’ perceptions regarding their needs, and challenges faced by them at various steps of the supply chain of the program, (c) To explore the key entry points of intervention at different stages of the supply chain to strengthen the program and diversify the foods/meals given under the program.

Target group: Partners at the State and District level-UNICEF, State Mother NGO, District NGO.

Introduction

Hello, I am ………………………………. from AIIMS, Bhopal. I am part of the NECCTAR trial research team exploring the current status of the THRs being provided in your community. We want to understand the supply chain of the program by finding out where the raw ingredients are obtained from, the manufacturing and processing involved, the distribution of the prepared THR to the Anganwadi Centres (AWCs), and final delivery to the beneficiaries. Along with this, we want to know if any communication strategies for nutrition education are being used in your community. We wish to find out ways of strengthening this program to improve the health and nutritional status of the community. The purpose is to strengthen and improve the program modalities leading to diversity in the diets of the beneficiaries and making them food secure. The final goal is to reduce malnutrition in young children.

This is just a conversation, and there are no right or wrong answers. If you are okay, I will be writing notes, and if you agree, I will also use this recorder for recording our conversation, so that I don't miss things. The interview will take around 30 minutes. Do you agree and consent to the interview?

1. Yes, 2. No

If consent is given by the participant, proceed with the interaction/interview.

1. Stakeholder information

**Table 8:** Stakeholder information

SN	Item		SN	Item	
1.1	State		1.2	District	
1.3	Respondent name		1.4	Organization name	
1.5	Designation		1.6	Area of operation	State District

2. General information about the organisation and its function

2.1. May I request you to tell us about how your organization participates and contributes in the ICDS/WCD department and health department activities? Special focus on the nutrition and community-related activities.

Probe: activities, focus areas, departments collaborating, mode of participation, specific contributions in nutrition and health activities.

3. General information about the ICDS programme and the Take-Home Ration (THR).

3.1. May I request you to tell us about the special strategy and efforts targeted at child nutrition under the ICDS program in the state and/or the select district (study district name)?

Probe: enrollment of beneficiaries, coverage for nutrition services, any special financial package, special effort, any CSR activity, any community processes.

3.2. May I request you to tell us about the strategy, decision-making, and guideline development for Take-Home Ration (THR) products, preparation and supply in the state and select district (study district name)?

Probe: products, composition, suitability for beneficiaries, any special adaptation/modification, manufacturer(s), source of raw materials, quality check and certification, packaging and labeling, supply.

3.3. In your opinion, how are the beneficiaries/households and community accepting and utilizing the THRs supplied under the ICDS program? What are the possible reasons?

Probes: acceptance (perceived quality and benefit, sociocultural suitability), utilization (use for children, use by other family members, use for other purposes), possible reasons for use and/or non-use.

3.4. In your opinion, what are the challenges related to the THR production, procurement, supply, and acceptance by beneficiaries? How can these be addressed?

Probes: THR related (quality, ingredients, preparation, packaging), supply and distribution (quantity, frequency, regularity, storage, wastage), household acceptance and use.

3.5. May I request you to tell us how the ICDS and nutrition service-related activities are monitored and supervised? What are the challenges faced/experienced, and how are these being addressed?

Probe: who supervises/monitors, schedule or frequency, activities done, quality, feedback, factors influencing and challenges, modalities or efforts to address them. 

4. Information about community and household IYCF practices

4.1. In your opinion, what activities have been undertaken or efforts made to improve the household-level IYCF practices? What have been the experiences with such efforts?

Probe: efforts to improve complementary feeding, dietary diversity for children, challenges, and lessons.

4.2. In your opinion, what are the challenges related to complementary feeding in young children? How could these be addressed? Who all can contribute?

Probe: challenges, person/group who could contribute, how?

5. Information about Social and Behaviour Change Communication (SBCC) 

5.1. May I request you to tell us about the overall communication strategy and actions being adopted under the ICDS program related to the young child feeding and THR use?

Probe: any specific communication strategy, campaign, targeting nutrition, THR or any other, use of job aids/tools by the ICDS team at different levels.

5.2. In your opinion, what efforts have been made or are being made for capacity building of the AWC and/or ICDS teams in delivering the nutrition and health education activities? What are the potential influencing factors? How could these challenges be addressed?

Probe: AWC team’s competence and confidence, IEC/BCC/SBCC materials and/or tools/job aids (content, local culture and language appropriateness, channel), training methods, influencers (positive and negative), possible modalities to address.

6. Information about coordination, community engagement, and accountability

6.1. May I request you to tell us about the coordination and collaboration between WCD and health departments for nutrition and health services delivery, including the THRs? What coordination mechanisms are in place?

Probe: roles played and contributions, coordination mechanisms and platforms, appropriateness, challenges, and how addressed.

6.2. May I request you to tell us about the support and contribution by other departments, persons, groups, or organizations for the nutrition and health activities in the state and select district? If yes, how?

Probe: who participate/contribute (community/panchayat/Jaanch Committee/ Mother’s Committee/ NGO/SHG/CBO/teachers/ others persons/organisation), mode of participation, schedule or frequency, challenges, and how addressed.

6.3. In your opinion, what are the challenges experienced related to the community engagement and participation in ICDS services in the state and select district? What are the potential influencing factors? How could these challenges be addressed?

Probe: challenges, positive influencers, negative influencers, reasons, person/group who could contribute, how?

7. Closure

7.1. Before closing the interaction, would you like to suggest anything that could improve the nutrition and health service delivery by the ICDS team?

We thank you for your critical contribution.

Interview guide-6

Manual of Procedures and Group Discussion/ Interview guide for stakeholder mapping in the Take-Home Ration (THR) program

Objectives of the tool: (a) To map the supply chain of the Take-Home Ration (THR) as a part of the Supplementary Nutrition Program (SNP) under Integrated Child Development Services (ICDS) and to identify key actors involved in the planning and implementation of the program, (b) To understand their role in each step of the THR supply chain, their link with each other and their influence on planning and implementation of the program.

Stakeholder to be contacted: (a) Policy level: Key people from the Ministry of Women and Child Development (Potential officials- Deputy director, CDPO, Assistant child development officer); (b) Implementation level: Supervisor, Anganwadi worker, Anganwadi helper, Panchayati Raj Institution (PRI) members.

Criteria for Selection: (a) Individuals involved in a THR supply chain stage, (b) Stakeholders from policy and implementation levels, to be able to map the entire supply chain and elaborate on the various key actors involved at supply chain stages.

Logistics: A quiet room with a large flat surface, e.g., an empty table/ floor. Materials: (1) Chart paper, (2) Markers, (3) Post-it notes, (4) Coins, (5) Recorder. Total Duration: 1 hour.

Introduction (5 min):

Hello, I am ………………………….. from AIIMS Bhopal, India. I am part of the NECCTAR trial research team exploring the current situation of the THRs being provided in your community. We want to understand the supply chain of the program and the key actors involved in the various stages of the supply chain and the planning and implementation of the THR component of SNP-ICDS. This will be done by finding out where the raw ingredients are obtained from, the manufacturing and processing involved, transport and distribution of the prepared THR to the Anganwadi Centres (AWCs) and final delivery to the beneficiaries.

Purpose of this group discussion/ interview:

The Integrated Child Development Services (ICDS) scheme is one of the flagship programs that aims to improve the health and nutritional status of the vulnerable groups of the population, such as children, pregnant, and lactating women. The ICDS involves a network of people who influence the proper functioning of this program. These range from policymakers to people who implement this program to the beneficiaries. The role of each of these key people and their interactions with each other significantly impact the functioning of the program.

We have come to you as you are a key functionary or a key person who can share important information about the planning and implementation of this program. Through this group discussion/ interview we want to map how the food given as part of supplementary nutrition program (SNP) under ICDS (Take home ration (THR)), flows from the production units to the beneficiaries, key people involved at each step, their interaction with each other, and what influence do they have in planning and implementation of this program and their perceived goals.

Instructions for the facilitator/ interviewer: (a) Explain the research team’s affiliation and study aim, (b) Ask the participants to introduce themselves and their role in the program, (c) Participant Briefing: Explain the study, purpose of the activity, and obtain written informed consent, (d) Obtain written informed permission before audio recording the session, (e) Define Purpose and Objectives: Ensure the study team and participants understand the purpose of using the NET Mapping tool.

Steps of tool implementation: Step 1 - Mapping the Supply Chain (10 minutes), Step 2 - Stakeholder mapping/ Identifying Key Actors (10 minutes), Step 3 - Identifying Roles (10 minutes), Step 4 - Linking Actors (10 minutes), Step 5 - Assessing Influence (10 minutes).

Questions:

1. What are your roles and responsibilities in THR supplied/prepared in the Anganwadi centers through ICDS in your district? (3 min); 2. What all food items are given as part of THR?

Probe: (a) Blended premix, (b) Whole foods, (c) Any other             

Instructions for the facilitator/ interviewer: (1) Ask participants to share the names of all the THR foods provided under SNP-ICDS. Then, ask for details on the quantities and frequencies of the THR foods provided, along with the beneficiaries, (2) If decentralized manufacturing of THR is happening, then capture all the raw ingredients procured for its manufacture.

Mapping the supply chain of Take-home ration (THR) under SNP and key actors involved at each step

Step 1: Mapping the supply chain of Take-home ration (THR) (10 min):

3. According to your personal experience and knowledge, how does the Take-home ration (THR), such as Blended premix, etc., provided for children under 3 years of age, pregnant and lactating women under the SNP-ICDS move through different stages, i.e., from the production unit to beneficiaries.

Probe: (a) Where is the THR prepared? (b) How does THR flow through different stages, i.e., from the production unit to beneficiariesHow is it transported to the Anganwadi Centres (AWCs)?

Probes: Please tell us how things are happening currently in your village/district. Is the manufacturing of THR centralized or decentralized?

Instructions for the facilitator/ interviewer: (a) Ask participants to describe how THR flows from raw material procurement to final delivery. Probe continuously to mark all the supply points, (b) Create a flow map on the chart paper to outline major supply points from procurement, production, transportation, to distribution, (c) If decentralized manufacturing of THR is happening, then map the supply chain points involved for the procurement of all the raw ingredients for the manufacture.

Step 2: Mapping the key actors in the supply chain of THR (10 min):

4.1. Who are the key actors involved at each step from the procurement of raw material to production, transport, and finally distribution of the THR through AWCs in your district?

List the actors at all steps of the supply chain. Probe: Actors include individual people, organizations, networks of people, etc., who hold a position or have some roles and responsibilities towards the implementation of the program.

Instructions for the facilitator/ interviewer: (a) Use the stick-on notes and probe participants to identify actors in each supply point. Write one actor in each note and place them around on the large sheet in front of them, (b) Give participants 10 min to identify actors. After this, use the actor’s checklist below to check if there are parts of the supply chain that are completely missed by participants. If that’s the case, prompt participants to consider these stages too, (c) Prompt the participant on each stage: "Are there any actors involved in the stage that are not captured yet?”, (d) Give participants a 5-min gentle reminder to finalize their list, (e) Use the actor checklist (e.g., fund approvers, transporters, quality controllers) provided in the tool to fill gaps, (f) Keep in mind that if participants want to add more actors later, they can do it anytime.

Actors' checklist:

4.2. Blended Premix: Flow of food from the production unit of blended premix to the AWCs. Who are the actors involved in: (a) Approving and releasing of funds, (b) Procurement of raw material for blended premix, (c) Quality checking of the raw material, (d) Manufacturing/production, processing, and packaging of blended premix (labeling, packaging material), (e) Quality check of processed packets, (f) Informing the production unit about the quantity required (demand generation/ raising an indent), (g) Transportation of stocks, (h) Middle point between production unit and anganwadi center (if any).

4.3. Who are the actors involved in overall planning and making decisions on: (a) Budget allocation for the SNP-ICDS and specifically for THR, (b) Planning of types of food products given as THR, and quantity (packets/amount) to be given, (c) Planning of supply chain logistics and management: (a) Selection of production unit, (b) Storage, (c) Transportation, (d) Overall network of supply within the district.

Step 3: Identifying Roles (10 minutes)

5.  As per your opinion, what is the main role of each actor? (10 min)

Here are some examples to probe the role of specific actors: (a) Process (P): e.g., timely delivery of foods, quality of the food delivered, smooth functioning of the program, (b) Cost (C): minimizing costs, acquiring funding, (c) Health and Nutrition (H): ensuring the overall health and nutritional status of the beneficiaries, (d) Probe: Some actors may be neutral and not share any of these roles. Some actors may have more than one of these roles.

Instructions for the facilitator/ interviewer: Prepare in advance a stick-on note with the role and stick it next to the stick-on note with the key actor’s name on the chart paper.

Step 4: Linking Actors (10 minutes)

6.  How are the actors involved in the supply chain of THR linked with one another? (10 mins)

Probe: Link in terms of flow of food, funding, and information. (a) Flow of food refers to the way the food commodities that are procured and distributed move across different actors, (b) Flow of funding refers to how the budget necessary for the functioning of the programme is issued, approved, released, and moved across different actors, (c) Flow of information refers to how information necessary for the functioning of the programme, such as information regarding requisition of commodities (quantity, type of food, demand generation/ raising indent for THR), quality control (feedback mechanism), and information for technical support (communication channels), moves across different actors.

Probe: We are not looking for the protocols, but how these linkages are working as per your personal experience. Ask for specific examples that illustrate some of the interactions among the actors.

Probe for group interviews if participants have differential opinions about a linkage: Can you further explain what you mean by this link? Can you provide some specific examples of an interaction between these two actors that you have previously observed?

Instructions for the facilitator/ interviewer: Keep the stick-on notes, colour pens etc., ready and pre-assign specific colours for specific aspects. Remember to use the same colours of coins and stars for rating purposes also. (a) Green: Food flow. (b) Blue: Information flow. (c) Red: Funding flow. 

Probe the participants to guide you to link the actors using arrows indicating the direction of the link and colours indicating the type of link (flow of funding-red, flow of food-green, flow of information-blue). If there is a mutual exchange, the arrow can have two heads.

Step 5: Assessing Influence (10 minutes)

7.  How much influence or power does each actor have with respect to:

7.1. Planning and shaping decisions, for example on: (a) How much budget is to be allocated per beneficiary for THR? (b) Which food products are to be given as part of THR, (c) Logistics and supply chain management of THR: (a) Selection of production units, (b) Storage, (c) Transportation and supply to different AWCs of the villages.

7.2. Implementation, for example: (a) Ensuring smooth flow of funds, (b) Quality assurance: blended premix, whole foods, (c) Ensuring smooth transportation and supply of THR across the supply chain, (d) Distribution of the THR to the beneficiaries in the required quantity according to the norms

Instructions for the facilitator/ interviewer: (a) For each aspect of the THR supply (such as the flow of fund), ask the participants to suggest which key actors have an influence/ say on that specific aspect, (b) Then, ask the participants to rate each actor’s influence from 0 to 5. Then, stack specific colour-coded coins for rating the influence for different aspects on the side of the stick-on note for a specific actor, (c) After the participant finishes, verbalize what you see, starting with the actors with the higher influence, and ask the participant to expand on the type of influence (in terms of their specific role) different actors have, (d) Allow participants to modify their rating (in terms of the coins assigned) if they want during this process, (e) You may also use specific colour-coded star ratings to assess the level of influence. Ask for influence on different aspects individually and record accordingly using a rating from 0 to 5, (f) Please inform the participants that by influence, we do not refer to the formal hierarchy of positions. (e.g., Actors at a lower level of the hierarchy might play a more important role in ensuring the planning and implementation of the SNP-ICDS).

Probes for further discussion: (a) I see that this actor has the highest influence. Why do you think that is? Where does their influence come from? Are they neutral or supportive or have conflicting interests? (b) You say that these actors have the same level of influence. What happens if they disagree? Is their influence based on the same grounds? Does it have the same range? (c) Are the actors neutral or supportive or have conflicting interests? (d) You have linked this actor to many others, but you say they don’t have much influence. Why do you think that is?

Probe for group interviews if participants disagree about the level of influence: Why do you think this actor has a lot of/little influence?

Closing: (5 min). Thank you for participating. Anything else to add etc.

Data Recording: (a) Record the session using an audio recorder (with participant consent), (b) Take photographs of completed maps after each activity for documentation, (c) Analyze maps to: (1) Understand the current THR supply chain. (2) Highlight key actors involved at each stage and their influence, (d) Collate all the supply chain maps from the total number of NET-mapping activities conducted. Based on all the supply chain maps, prepare a comprehensive map and a list of all stakeholders involved in the THR supply chain.

DOs: (1) A trained research team should administer the NET mapping tool. The team should understand the context of the study and the purpose of the tool, (2) Practice facilitation using the script to reduce hesitations or biases, (3) Establish rapport with participants by introducing yourself and explaining the purpose of the activity, (4) Use active listening techniques, such as nodding and summarizing key points, to show engagement, (5) Use simple language to explain each step of the NET-Mapping process, (6) Encourage active participation from all stakeholders, (7) Maintain a neutral tone to encourage open and honest participation, (8) Handle sensitive information with discretion and maintain confidentiality, (9) Prepare all materials in advance and test the audio recorder before the session, (10) Facilitate the discussion and probe to ensure all relevant actors at various stages are identified. A key objective of the tool is to conduct stakeholder mapping to identify all relevant key actors involved at each stage of the THR supply chain, (11) Encourage participants to provide insights beyond the mapped roles to uncover unknown dynamics, (12) Document the activity with audio recordings (with consent), (13) Validate the completed map with participants to confirm accuracy and take clear photographs of the final map.

DON’Ts: (1) Don’t interrupt participants while they are sharing their inputs, (2) Avoid leading questions that may bias participant responses, (3) Don’t assume any roles or linkages without participant confirmation, (3) Don’t rush through the steps; allow enough time for discussions, (5) Do not let dominant participants monopolize the discussion; use gentle redirection techniques, (6) Avoid using technical jargon or language that may confuse participants, (7) Don’t record the session without explicit consent from participants, (8) Don’t disclose participants’ responses or sensitive findings outside the research context.
